The article "Analysis of Carotid Ultrasound Screening of High-Risk Groups of Stroke Based on Big Data Technology" was retracted in 2023. Reasons: signs of a paper mill; compromised peer review; unreliable results or conclusions.

# Analysis of Carotid Ultrasound Screening of High-Risk Groups of Stroke Based on Big Data Technology

**DOI:** 10.1155/2022/6363691

**Published:** 2022-01-25

**Authors:** Jiankang Guo, Yanhong Bai, Minxia Ding, Lisha Song, Guo Yu, You Liang, Zhigang Fan

**Affiliations:** ^1^Department of Ultrasound Medicine, 3201 Hospital, Shanxi 723000, China; ^2^Department of Oncology, 3201 Hospital, Shanxi 723000, China

## Abstract

In order to understand detection of carotid atherosclerosis in the screening of high-risk stroke populations in a certain area of China, we have analyzed related risk factors of CAS. In accordance with the requirements of the “2015 Technical Plan for the Screening and Intervention Projects for High-Risk Stroke Populations,” a cluster sampling method was used to select 4532 (number of screened persons from 2015 to 2021) permanent residents over 41 years old (一) in Shaheying Town, Liulin Town, Chenggu County, Hanzhong City, Shaanxi Province, and Da'an Town, Ningqiang County, and nearby communities are selected as the screening targets. We screened out high-risk groups of stroke based on big data technology and understood the detection of CAS. According to the screening results of big data technology, it was divided into two groups: CAS group and non-CAS group. The basic information, medical history, personal lifestyle, physical examination, and laboratory examination results of the two groups were classified and counted. The measurement data such as age and waist circumference of the two groups were tested by two independent samples, and the count data of gender, stroke history, hypertension, and other data were tested by the *χ*^2^ test of the four-table data, and the logistic regression model was used to analyze the risk factors for CAS of population at high risk of stroke. The results proved the following: (1) Among the 4532 screeners, 865 cases were screened out of the high-risk population of stroke, with an average age of (58.5 ± 8.3) years, mainly 59 to 68 years old, accounting for 43.8%, and the male-to-female ratio was 1.6 : 1. (2) The detection rates of CAS, intimal thickening, plaque formation, and stenosis among high-risk groups of stroke were 55.5%, 10.2%, 52.2%, and 32.6%, respectively. (3) Among the high-risk groups of stroke, CAS patients have a history of stroke, the proportion of hypertension, age, total cholesterol, and low-density lipoprotein cholesterol levels that are higher than those in the non-CAS group, and the difference is statistically significant. (4) Logistic regression analysis shows that age, diabetes, and low-density lipoprotein cholesterol are independent risk factors for CAS in the high-risk population of stroke in this area.

## 1. Introduction

Stroke has become the leading cause of death and disability among Chinese residents. There are currently about 70 million stroke patients in my country, about 2 million new strokes occur every year, and about 1.88 million people die from stroke each year. Chinese people who die from stroke each year account for 22.45% of the total deaths [1]. Therefore, stroke seriously threatens human health. According to clinical experience at home and abroad, stroke is preventable and controllable. Effective intervention for the risk factors of stroke can not only reduce the incidence of stroke, but also reduce various burdens caused by stroke. There are many risk factors that affect stroke, which can be divided into nonintervention and interventionable. Among them, nonintervention factors include age, gender, race, genetic factors, etc., and intervention factors include improper lifestyle, hypertension, hyperlipidemia, diabetes, atrial fibrillation, and asymptomatic carotid atherosclerosis. Studies have shown that CAS is an independent risk factor for stroke [2]. As an important blood supply route for the brain, the carotid artery can reflect the degree of atherosclerosis of the arteries throughout the body. It has the advantages of superficial location and easy detection. Lee et al. [3] showed that the carotid artery intima-media thickness is an important indicator of arterial wall disease. In 2007, Lorenz [4] et al. conducted a 5.5-year follow-up study of 37, 197 people and found that for every 0.1 mm increase in CIMT, the risk of stroke will increase by 13% to 18%. Carotid ultrasound measurement of CIMT and carotid plaque can help determine the degree of CAS. It has the advantages of noninvasive, safe, low-cost, convenient, and repeatable inspection. Therefore, the discovery of CAS through ultrasound is of great significance in predicting stroke. CAS is a pathophysiological process caused by a variety of factors. Many studies have shown that CAS is closely related to many risk factors such as age, gender, ethnicity, multiple chronic diseases, bad living habits, snoring, etc. It is also closely related to the Hcy, C-reactive protein, uric acid, fibrinogen, tumors, polyarteritis, iron deficiency anemia, antithrombin III reduction, and other factors. However, from the perspective of medical treatment and disease treatment, attention should be paid to the common risk factors that have been identified. My country has gradually entered an aging society. The high incidence of cerebrovascular diseases in the elderly will surely become the focus of our prevention and treatment. At present, cerebrovascular diseases are becoming younger. Therefore, it is necessary to strengthen the screening of CAS for middle-aged and elderly people, and to deal with the many causes of CAS. Early comprehensive intervention of various risk factors to delay the occurrence and development of CAS is of great significance to the prevention and treatment of stroke [5].

(二) In this paper, we have used big data technology to sample and screen permanent residents over 40 years of age in Shaheying Town, Liulin Town, Chenggu County, and Da'an Town, Ningqiang County, Hanzhong City, Shaanxi Province, to screen out high-risk stroke populations to understand the CAS detection status of local high-risk stroke populations and related risk factors. Likewise, we have provided information for the prevention and treatment of CAS in the region practical scientific basis. It is hoped that through the prevention and treatment of CAS, the incidence of stroke due to CAS can be reduced.

The remaining paper is organized as follows: in the subsequent section, we have provided a comprehensive literature review of those mechanisms which are closely linked to the proposed methodology. In Section 3, the proposed method along with selection and rejection criteria for various groups is presented. Experimental results and observations are provided in Section 5 of this manuscript which is followed by a comprehensive and generalized discussion. Finally, concluding remarks along with future directives are provided in the last section.

## 2. Related Work

Atherosclerosis is a lesion characterized by the deposition of subintimal lipids, fibrosis, and atherosclerosis, which are mainly involved in the large and middle arteries, which in turn causes the vascular wall to become hardened and vascular. The cavity is narrow, leading to secondary cardiovascular and cerebrovascular diseases. As a part of the systemic artery, the carotid artery can reflect systemic arteriosclerosis. CAS has obvious characteristics of AS. Therefore, the risk factors of CAS are consistent with AS. The formation, occurrence, and development of CAS are related to a variety of risk factors. It not only includes traditional risk factors such as age, gender, race, smoking, alcoholism, obesity, high blood pressure, hyperlipidemia, diabetes, etc., but also includes homocysteine, uric acid, C-reactive protein, etc., which have only been gradually recognized in recent years, and they are all closely related to CAS.

With the increase of age, the exposure of patients to other risk factors also increases, especially the elderly over 65 years old often have target organ damage caused by cardiovascular and cerebrovascular diseases, and the two play a common role in the development of CAS [6]. Most clinical studies have shown that the incidence of CAS in men is higher than that in women [7–9], which may be related to poor lifestyles such as high blood lipids, coronary heart disease, and smoking and alcoholism in men. A meta-analysis [10] showed that 393 participants lost an average weight of 16 kg during an average follow-up of 20 months, and the average change in carotid artery intima-media thickness was −0.03 mm. Therefore, in obese people, weight loss was not only positive with the reduction of CIMT. Correlation can also reduce the risk of cardiovascular and cerebrovascular events. Relevant studies have shown [11, 12] that high levels of active oxygen and active nitrogen in smokers make LDL-C more oxidizable, thereby accelerating the process of AS. The results of Chen et al. [13] showed that smoking can cause a decrease in serum folate and superoxide dismutase levels, an increase in homocysteine content, and oxidative damage to the blood vessel wall, which further promotes the formation and progression of AS.

In 2010, Xie et al. [14] conducted a study on 14,618 Chinese people over 35 years old and showed that among men, alcohol intake was correlated with peripheral AS, and alcohol consumption of less than 60 g/day was negatively correlated with ankle-brachial index. And when the alcohol consumption exceeds 60 g/day, it is positively correlated with the ankle-brachial index; the study did not find a correlation between peripheral AS and female alcohol consumption. In the same year, Zyraix et al. [15] conducted a study on healthy people aged 30–70 years and showed that among men, daily alcohol consumption was positively correlated with CIMT, while this correlation was not significant among women. In 2012, Xie and his team [16] surveyed 13,037 Chinese people and found that drinking in the Han population was correlated with CAS, while a small amount of drinking was negatively correlated with CAS. The latest research progress has shown [17] that drinking has positive and negative effects on cardiovascular and cerebrovascular diseases, and the mechanism of different effects may be related to the amount, duration, and drinking style of alcohol.

Studies believe that [18, 19] lack of exercise is an important risk factor for CAS and carotid plaque formation. Aerobic exercise can prevent and control the occurrence and development of CAS. The mechanism is as follows: (1) reduce TC, TG, and LDL-C levels to regulate lipid metabolism; (2) improve vascular endothelial dysfunction; (3) strengthen the body's antioxidant activity ability to delay the occurrence and development of CAS [20]. Recent studies have shown [21] that only moderate-intensity aerobic exercise produces more nitric oxide than reactive oxygen species and increases vascular endothelial function. Low-intensity aerobic exercise has no benefit, but high aerobic exercise is harmful. Lannuzzi et al. [22] confirmed that a low-calorie diet is beneficial to improve the thickness and hardness of the carotid artery intima in obese children, and for the first time demonstrated that a low-glycemic index diet can improve insulin sensitivity in obese children. Leite et al. [23] believe that a low-carbohydrate diet can not only reduce weight and lipid deposition, but also prevent the accumulation of oxidized low-density lipoprotein and reduce the production of inflammatory cytokines in the vessel wall, thereby preventing AS. Studies have shown [24] that dietary fresh vegetables and fruits can prevent the occurrence of early CAS. Proietti et al. [25] have shown that frequent consumption of vegetables and fruits is negatively correlated with CAS, while frequent consumption of milk or yogurt is positively correlated with carotid plaque formation. However, Casalnuovo et al. [26] believe that medium-chain fatty acids, including dairy products, can reduce the accumulation of visceral fat and subcutaneous fat, improve lipid metabolism, and prevent the occurrence of AS. The relationship between dairy products and CAS needs to be further studied, but high-salt, high-fat, and high-sugar diets can aggravate CAS by causing hypertension, hyperlipidemia, and hyperglycemia.

It proposed that the incidence of CAS in hypertensive patients is positively correlated with blood pressure variability. Hypertension can affect the function of vascular endothelial cells, increase the permeability of the vascular wall, facilitate the deposition of lipids in the vascular wall, cause hemodynamic changes, activate the inflammatory response, enhance the coagulation mechanism and the susceptibility to AS, and ultimately lead to and promote the formation of AS [27]. Diabetes is an important risk factor for CAS, which not only accelerates the natural process of CAS, but is also a predictor of the progression of CAS. Tropeano et al. [28] have shown that hyperglycemia is an independent risk factor for CIMT thickening in patients with essential hypertension, regardless of whether the patient is type 2 diabetic or in the early stage of impaired fasting blood glucose. Dyslipidemia is one of the important risk factors for AS. High levels of total cholesterol, low-density lipoprotein cholesterol, and triglycerides in serum can not only directly lead to the formation of AS through lipid deposition and other mechanisms, but also promote oxidative stress, produce inflammation, secrete cytokines, and activate coagulation factors. Increase the risk factors of AS, thereby promoting the occurrence and development of AS.

CAS is a chronic pathophysiological process caused by many factors. Its pathogenic factors include not only uncontrollable risk factors such as age but also controllable risk factors such as hypertension. However, the pathogenic mechanism of some factors is not clear, and the research results are not consistent. Therefore, it is necessary to further deepen the research and exploration of the mechanism and pathogenic risk factors of CAS to provide a stronger theoretical basis for the prevention and treatment of CAS. At the same time, comprehensive measures must be taken to prevent and control controllable risk factors in order to effectively reduce and prevent the brain occurrence and development of vascular disease.

## 3. Materials and Methods

### 3.1. General Materials

#### 3.1.1. Research Object

Relying on the “2015 stroke prevention and screening project of the national health and Family Planning Commission,” we used big data technology to cluster screen the permanent residents over 40 years old in shaheying Town, Liulin Town, Chenggu County, and Da'an Town, Ningqiang County, Hanzhong City, Shaanxi Province, including those living in the local area for more than half a year. According to the “Technical Specifications for Stroke Screening and Prevention and Treatment,” the high-risk populations of stroke were screened out according to the screening criteria for high-risk populations, and those who had perfected carotid artery color Doppler ultrasound were selected as the target population. A total of 704 cases were collected. According to the results of carotid artery color Doppler ultrasound, the target population is divided into two groups according to whether there is CAS: CAS group and non-CAS group.

#### 3.1.2. Inclusion Criteria

Residents who are over 41 years old and have local household registration meet the high-risk population of stroke in the “Stroke Screening and Prevention Technical Specifications” promulgated by the National Health and Family Planning Commission's Stroke and Screening Prevention Engineering Committee and improve the carotid artery color Doppler inspection.

#### 3.1.3. Exclusion Criteria

Exclusion criteria are those who do not meet the above inclusion criteria and have undergone carotid endarterectomy, vascular bypass, or interventional therapy before this survey.

### 3.2. Proposed Methodology

#### 3.2.1. Screening Information

General information of screeners through big data technology is collected: name, gender, household registration, ethnicity, and export; basic information such as date of birth, marital status, occupation, education level, and personal average annual income; lifestyles such as smoking, drinking, exercise habits, dietary habits, family history of stroke, history of stroke, heart disease, hypertension, diabetes, dyslipidemia, and other past history and drug control status.

#### 3.2.2. Judgment Criteria for High-Risk Groups of Stroke

According to the “Stroke Screening and Prevention Technical Specifications” promulgated by the National Health and Family Planning Commission's Stroke Screening and Prevention Engineering Committee, the following 8 risk factors are risk assessed, as shown in Tables 1 and 2.

#### 3.2.3. Carotid Artery Ultrasonography

The ultrasound medical department of our hospital (3201 hospitals) sent two professionally trained doctors to conduct neck vascular ultrasound examination for people at high risk of stroke, use Philips color Doppler ultrasound diagnostic instrument for diagnosis, and select 3∼12 MHz broadband linear array probe and 1∼5 MHz convex array probe for joint inspection. Take the supine position, fully expose the neck of the examination side, and observe the IMT, plaque, and stenosis of the neck blood vessels.

In this study, the CIMT thickening ≥1 mm was used as a sign of the beginning of CAS. The definition of IMT and plaque is as follows: (1) IMT < 1.0 mm is normal, IMT is 1.0 mm ≤ IMT < 1.5 mm, and IMT is thickened; (2) the lumen intima and media are locally irregularly thickened, protruding to the cavity. Within, IMT ≥ 1.5 mm is defined as plaque. Specific contents of cervical vascular ultrasound examination are (1) thickening of IMT: the distal part of the common carotid artery; (2) plaque: the bilateral common carotid artery, internal carotid artery, subclavian artery, and vertebrae arteries; the number is to record the number of plaques in each segment and sum; and (3) stenosis: the sites are bilateral common carotid arteries, internal carotid arteries, subclavian arteries, and vertebral arteries; grades are mild, moderate, severe, and occluded. The evaluation criteria at all levels are as follows [29]: mild—the stenosis rate is normal or <50%, the blood flow at the stenosis site has no obvious change, the arterial lumen becomes slightly smaller, and the PSV and EDV have no obvious change or increase slightly; moderate—the stenosis rate is 50–69%, the flow velocity in the arteries becomes thinner, the PSV and EDV are accelerated, and the PSV and EDV at the distal end of the stenosis are reduced; severe—the stenosis rate is 70–99%, the blood flow bundle in the artery is obviously thinned, and the PSV and EDV in the stenosis are obvious; speedup—PSV and EDV at the distal end of the stenosis significantly slow down; and occlusion—there is no blood flow signal in the vessel lumen.

#### 3.2.4. Criteria for CAS-Related Risk Factors

1. Frequent heavy drinking: Liquor is 3 times a week or more, and each time is more than two tales
2. Stroke: A stroke/TIA is clearly diagnosed in a hospital above the second level
3. For risk factors such as smoking, hypertension, diabetes, dyslipidemia, and stroke genetics, refer to Table 1

#### 3.2.5. Quality Control

This study conducted unified training for medical personnel participating in on-site questionnaire surveys, physical examinations, blood collection, blood specimen submission, laboratory testing, carotid artery color Doppler ultrasound examinations, and data entry and carried out strict quality control, expert verification, and correct errors in time. (五) The data are uploaded to the cerebrovascular disease big data platform of stroke prevention and Control Engineering Committee of National Health Commission (https://chinasdc.cn), and quality control is carried out by random inspection. For problematic data, the original records are verified and corrected. Expert of stroke prevention and Control Engineering Committee of National Health Commission evaluate the data reported directly from the Internet and feed back the evaluation results to achieve real-time monitoring of the quantity and quality of screening work.

## 4. Experiments and Results

### 4.1. Basic Characteristics of People at High Risk of Stroke

According to Tables 3 and 4, a total of 4800 questionnaires were screened, and 4532 were qualified, with a pass rate of 94.4%, which met the 85% sampling requirements of the National Health and Family Planning Commission's Stroke Prevention and Screening Project. (六) Among the 4532 screeners, there were 2995 cases in Shaheying Town and Liulin Town, 620 cases in high-risk groups of stroke, 1537 cases in Da'an Town, and 332 cases in high-risk groups in the district, 952 cases in total. There is no significant difference in the detection rate of high-risk groups in the two places. Among the high-risk populations initially screened, 87 cases failed to complete the carotid artery ultrasound examination. Therefore, the target population was 865, which was in line with the sampling rate of 85%. There are 865 high-risk groups of stroke, the age range is 41–83 years old, and the average age is (58.5 ± 8.3) years old, mainly 59–68 years old: 61.7% of males, 38.3% of females, and male-to-female ratio 1.6 : 1, male mainly; Han nationality accounted for 91.5%, and ethnic minorities accounted for 8.5%, mainly Han nationality: smoking 41.2%, drinking 25.8%, lack of exercise 48.5%, overweight 80.7%, stroke 18.2%, stroke family history 17.8%, and hypertension. The disease was 68.2%, diabetes was 20.4%, and dyslipidemia or unknown was 33.4%. Physical examination and laboratory indicators are average neck circumference (38.4 cm ± 3.4) cm, average waist circumference (93.1 ± 8.5) cm, average TG (2.1 ± 1.2) mmol/L, average TC (5.2 ± 1.1) mmol/L, the average LDL-C (3.5 ± 0.9) mmol/L, and the average HDL-C (1.1 ± 0.3) mmol/L which is shown in Figures 1 and 2.

### 4.2. Comparison of Carotid Artery Ultrasound Examination Results

#### 4.2.1. Comparison of Results of Arterial Ultrasonography of Different Genders

Among the high-risk population of stroke, the detection rate of CAS was 55.6% in men and 52.8% in women; the detection rates of CIMT thickening, plaque formation, and stenosis in men were 10.1%, 51.8%, and 29.8%, respectively, and the corresponding detection rates in women were 7.6%, 50.2%, and 34.3%, respectively. The detection rates of CAS, CIMT thickening, and plaque formation in men were higher than those in women, while the detection rate of carotid artery stenosis in women was higher than that in men. See Table 5 for details.

#### 4.2.2. Comparison of Results of Arterial Ultrasonography in Different Age Groups

The detection rates of CAS among high-risk groups of stroke in different age groups were 21.0%, 41.8%, 67.3%, and 84.0%, respectively, and the differences were statistically significant; CIMT thickening, plaque formation, and carotid artery stenosis were all in 41–50 years old. The detection rate is the lowest in the age group, and the detection rate is the highest in the age group over 70. There are significant statistical differences between the above groups which is shown in Figure 3. See Table 6 for details.

#### 4.2.3. Comparison of Non-CAS Group and CAS Group

Among the 865 high-risk groups of stroke, 385 cases (44.50%) were non-CAS, 480 cases (55.5%) were CAS, and most of them were CAS. The CAS group was divided into CIMT thickening and plaque formation. There were 29 cases of pure CIMT thickening, accounting for 6.00% of CAS, and 452 cases of plaque formation, accounting for 94.2% of CAS.

#### 4.2.4. Logistic Regression Analysis of the CAS Single Factor

In order to clarify the independent risk factors of CAS in this area, the independent variables were first screened out by univariate analysis. After a single factor logistic regression analysis, age, family inheritance of stroke, diabetes, stroke history, hypertension, TC, and LDL-C were selected as independent variables of the multivariate regression analysis, as shown in Table 7.

#### 4.2.5. Logistic Regression Analysis of CAS Multifactors

The selected independent variables were incorporated into a multivariate logistic regression analysis model. Through stepwise regression analysis, the risk factors of CAS in high-risk stroke populations were explored. The results showed that age, diabetes, and high LDL-C are the risk factors for CAS in high-risk stroke populations in the region. In independent risk factors, the difference is statistically significant; see Table 8 for details.

## 5. Conclusions

This paper uses big data technology to screen out 865 cases of high-risk stroke groups from 4532 screeners. CAS is an independent risk factor for stroke. Its occurrence and development process include CIMT thickening, plaque formation, stenosis, and occlusion. CAS is a chronic pathophysiological process caused by multiple factors. Its pathogenic factors include not only uncontrollable risk factors such as age, but also controllable risk factors such as hypertension, but the pathogenic mechanism of some factors is not clear. Therefore, we must not only pay attention to the process of CAS, but also pay attention to the risk factors that lead to the occurrence and development of CAS. Therefore, this project provides a theoretical basis for the early detection, prevention, and diagnosis of CAS through the analysis and research on the detection of CAS and related risk (七) factors in Hanzhong City, China. The basic characteristics of the high-risk population of stroke are 59–68 years old, male, Han nationality, a large number of overweight people, a high prevalence of hypertension, and a large proportion of abnormal blood lipids; TG and LDL-C are higher than the normal reference range, TC is at the upper limit of normal value, and HDL-C is at the lower limit of normal value. As we all know, age and gender are the most uncontrollable risk factors for stroke. Elderly men must be the key population for stroke prevention and treatment. The high-risk population for stroke in this study is mainly elderly men, which is consistent with a large number of literature reports. The local residents over 40 years old selected in this study are mainly the elderly over 60 years old. Their blood vessels tend to age, their nutritional intake increases with the improvement of their living standards, and they prefer a high-salt diet, lack of exercise, obesity, and other reasons. The prevalence of hypertension in high-risk groups of stroke is relatively high. The proportion of overweight and dyslipidemia among high-risk groups is relatively high, and TG and LDL-C are relatively high. Considering that the residents in this area are mainly like pasta and fried food, but the intake of vegetables and fruits is insufficient, the residents' life is relatively monotonous and there are few outdoor sports. In addition, the screening time is after the Spring Festival. During the Spring Festival, there may be factors such as excess nutrition and less activity, which is more conducive to weight gain and abnormal blood lipids.

## Figures and Tables

**Figure 1:** Age composition ratio of high-risk stroke population.

**Figure 2:** Gender composition ratio of high-risk stroke population.

**Figure 3:** Comparison of results of arterial ultrasonography in different ages.

**Table 1:** Judgment criteria for risk factors of stroke.

Risk factors	Judgment standard
Hypertension	Systolic blood pressure ≥140 or diastolic blood pressure ≥90 mm Hg or taking antihypertensive drugs
Heart disease	Atrial fibrillation or obvious irregular pulse
Smoking	At least 1 cigarette a day, for at least 1 week
Dyslipidemia	TG ≥ 2.26 or TC ≥ 6.22 or LDL-C ≥ 4.14 or HDL-C ≤ 1.04
Diabetes	Fasting blood glucose ≥7.0 mmol/L
Physical exercise	3 times a week or more, 30 minutes or more once
Significantly overweight	BMI≥26 kg/m^2^
Family inheritance	Family inheritance of stroke

**Table 2:** Judgment criteria for high-, medium-, and low-risk groups of stroke.

Crowd classification	Judgment standard
High-risk groups	3 or more risk factors or a history of stroke or TIA
Medium-risk groups	Less than 3 risk factors and suffer from chronic diseases
Low-risk groups	Less than 3 risk factors and no chronic diseases

**Table 3:** General information of people at high risk of stroke.

Item	Number of cases	Percentage
Sex (male)	534	61.7
Nationality (Han)	792	91.5
Smoking	356	41.2
Drinking	223	25.8
Lack of exercise	420	48.5
Overweight	698	80.7
Hypertension	590	68.2
Diabetes	176	20.4
Dyslipidemia	289	33.4
Stroke	157	18.2
Stroke inheritance	154	17.8

**Table 4:** Physical examination and laboratory indicators.

Item	Average and error range
Neck circumference (cm)	38.4 cm ± 3.4
Waist circumference (cm)	93.1 ± 8.5
TG (mmol/L)	2.1 ± 1.2
TC (mmol/L)	5.2 ± 1.1
LDL-C (mmol/L)	3.5 ± 0.9
HDL-C (mmol/L)	1.1 ± 0.3

**Table 5:** Comparison of results of arterial ultrasonography of different genders.

Item	Male *N* = 532	Female *N* = 333	*χ* ^2^	*P*
CAS	296	176	0.53	0.47
CIMT thickening	54	25	1.26	0.26
Plaque formation	276	167	0.17	0.68
Narrow	159	114	1.62	0.21

**Table 6:** General comparison of the non-CAS group and CAS group.

Item	Non-CAS *N* = 385	CAS *N* = 480	*χ* ^2^	*P*
Sex (male)	228	297	0.53	0.47
Nationality (Han)	349	442	0.09	0.76
Smoking	161	195	0.07	0.79
Drinking	105	119	0.62	0.43
Hypertension	229	362	20.5	0.00
Diabetes	59	118	9.3	0.00
Dyslipidemia	133	156	0.38	0.54
Stroke	41	118	22.8	0.00
Stroke inheritance	84	69	6.6	0.01

**Table 7:** Logistic regression analysis of the CAS single factor.

Risk factors	*B*	SE	*P*	OR	ORCI
Age	0.11	0.01	0.00	1.11	1.09∼1.14
Sex (male)	−0.11	0.16	0.47	0.89	0.66∼1.21
Nationality (Han)	−0.19	0.27	0.47	0.82	0.49∼1.39
Smoking	−0.04	0.15	0.79	0.96	0.71∼1.30
Drinking	−0.15	0.17	0.39	0.86	0.61∼1.21
Hypertension	0.74	0.16	0.00	2.09	1.52∼2.89
Diabetes	0.59	0.20	0.00	1.81	1.23∼2.65
Dyslipidemia	−0.10	0.16	0.54	0.91	0.66∼1.24
Stroke	1.01	0.22	0.00	2.75	1.80∼4.20
Inheritance	−0.51	0.20	0.01	0.60	0.41∼0.89
Neck (cm)	0.01	0.02	0.67	1.01	0.97∼1.06
Waist (cm)	0.01	0.01	0.46	0.99	0.98∼1.01
TG	0.11	0.06	0.07	0.90	0.79∼1.01
TC	0.22	0.08	0.00	1.24	1.07∼1.45
LDL-C	0.25	0.08	0.00	1.28	1.09∼1.50
HDL-C	−0.01	0.26	0.97	1.01	0.61∼1.67

**Table 8:** Logistic regression analysis of CAS multifactors.

Risk factors	*B*	SE	*P*	OR	ORCI
Age	0.11	0.01	0.00	1.11	1.09∼1.13
Diabetes	0.46	0.21	0.03	1.58	1.04∼2.40
LDL-C	0.25	0.09	0.01	1.29	1.08∼1.53

## Data Availability

The datasets used and analyzed during the current study are available from the corresponding author upon reasonable request.
